# Murepavadin, a Small Molecule Host Defense Peptide Mimetic, Activates Mast Cells *via* MRGPRX2 and MrgprB2

**DOI:** 10.3389/fimmu.2021.689410

**Published:** 2021-06-23

**Authors:** Aetas Amponnawarat, Chalatip Chompunud Na Ayudhya, Hydar Ali

**Affiliations:** ^1^ Department of Basic and Translational Sciences, School of Dental Medicine, University of Pennsylvania, Philadelphia, PA, United States; ^2^ Department of Family and Community Dentistry, Faculty of Dentistry, Chiang Mai University, Chiang Mai, Thailand; ^3^ Department of Oral Diagnosis, Faculty of Dentistry, Naresuan University, Phitsanulok, Thailand

**Keywords:** murepavadin, mast cells, MrgprB2, MRGPRX2, host defense peptides, antimicrobial peptides

## Abstract

*Pseudomonas aeruginosa* is a frequent cause of hospital-acquired wound infection and is difficult to treat because it forms biofilms and displays antibiotic resistance. Previous studies in mice demonstrated that mast cells (MCs) not only contribute to *P. aeruginosa* eradication but also promote wound healing *via* an unknown mechanism. We recently reported that host defense peptides (HDPs) induce human MC degranulation *via* Mas-related G protein-coupled receptor-X2 (MRGPRX2). Small molecule HDP mimetics have distinct advantages over HDPs because they are inexpensive to synthesize and display high stability, bioavailability, and low toxicity. Murepavadin is a lipidated HDP mimetic, (also known as POL7080), which displays antibacterial activity against a broad panel of multi-drug-resistant *P. aeruginosa*. We found that murepavadin induces Ca^2+^ mobilization, degranulation, chemokine IL-8 and CCL3 production in a human MC line (LAD2 cells) endogenously expressing MRGPRX2. Murepavadin also caused degranulation in RBL-2H3 cells expressing MRGPRX2 but this response was significantly reduced in cells expressing missense variants within the receptor’s ligand binding (G165E) or G protein coupling (V282M) domains. Compound 48/80 induced β-arrestin recruitment and promoted receptor internalization, which resulted in substantial decrease in the subsequent responsiveness to the MRGPRX2 agonist. By contrast, murepavadin did not cause β-arrestin-mediated MRGPRX2 regulation. Murepavadin induced degranulation in mouse peritoneal MCs *via* MrgprB2 (ortholog of human MRGPRX2) and caused increased vascular permeability in wild-type mice but not in MrgprB2^-/-^ mice. The data presented herein demonstrate that murepavadin activates human MCs *via* MRGPRX2 and murine MCs *via* MrgprB2 and that MRGPRX2 is resistant to β-arrestin-mediated receptor regulation. Thus, besides its direct activity against *P. aeruginosa*, murepavadin may contribute to bacterial clearance and promote wound healing by harnessing MC’s immunomodulatory property *via* the activation of MRGPRX2.

## Introduction

The emergence of multidrug-resistant bacterial infections poses a global public health threat that warrants urgent need for alternative therapeutic approaches (1). Host defense peptides (HDPs), previously known as antimicrobial peptides (AMPs), such as the cathelicidin LL-37 and human β-defensins are considered as promising antimicrobial agents (2–4). Recent evidence demonstrated that in addition to their direct antimicrobial activity, HDPs promote the recruitment and activation of various immune cells including mast cells (MCs), neutrophils, monocytes and lymphocytes (5–8). These HDPs also display angiogenic activity and contribute to wound healing (8, 9). However, many HDPs cause the lysis of erythrocytes and display cytotoxicity against a variety of cells (10, 11). In recent years, great strides have been made in optimizing HDPs to minimize their toxicity and to improve their stability, which can also modulate the immune system for therapeutic benefits (12, 13).

Mast cells (MCs) are multifunctional immune cells of hematopoietic origin that are found in vascularized tissues such as the oral mucosa, intestine, airway and the skin. MCs play an important role in host defense and promote wound healing (14–16). In addition to high affinity IgE receptor (FcϵRI), a subtype of human MCs (MC_TC_; contain both tryptase and chymase) expresses a G protein-coupled receptor (GPCR) known as Mas-related GPCR-X2 (MRGPRX2) (17, 18). This receptor is highly expressed in human skin MCs but is also present in lung and gut MCs but at lower levels (17, 19, 20). Mouse connective tissue MCs (CTMC; skin, nasopharynx and peritoneal) express MrgprB2 (ortholog of human MRGPRX2) (16, 21). Both receptors are activated by human and mouse HDPs (22–24). Studies with human MCs expressing MRGPRX2 and MrgprB2^-/-^ mice have strongly implicated these receptors in innate immunity and wound healing (15, 16). The major portal of entry for pathogen is the interface between host and external microenvironment such as the skin, nasopharynx, and peritoneum. MrgprB2-expressing CTMCs are found abundantly at these sites and contribute to host defense against bacterial infection through the release of MC-derived mediators and the subsequent recruitment of neutrophils (16). Furthermore, pharmacological activation of MrgprB2 at these sites results in decreased bacterial count and reduced disease severity *in vivo* (16).

*Pseudomonas aeruginosa* is a Gram-negative bacterium that often presents a therapeutic challenge due to its ability to form biofilms and to display antibiotic resistance (25, 26). Zimmerman et al. (27), utilized a topical *P. aeruginosa* infection model and demonstrated that MCs contribute to both bacterial elimination and promote wound healing. However, they found that culturing MCs infected with *P. aeruginosa in vitro* is insufficient to eliminate bacteria unless they are co-cultured with keratinocytes. MC mediators released in response to *P. aeruginosa* infection results in the secretion of HDPs such as mouse β-defensin-14 (Defb14, ortholog of human β-defensin-3) from keratinocytes (27). These findings suggest that MC-derived mediators confer protective immunity through the promotion of endogenous HDP secretion, which in turn, directly kill the bacteria and restrain the infection (27).

Protegrin-1 is a HDP that was originally purified from porcine leukocytes (28). We have recently shown that protegrin-1 activates human MCs *via* MRGPRX2 (29). However, small molecule HDP mimetics have a number of advantages over natural HDPs because of their superior stability, bioavailability, and reduced toxicity (30, 31). Moreover, several approaches have been used to increase hydrophobicity and membrane activity of HDP mimetics (32). Murepavadin is a lipidated protegrin-1 mimetic, (also known as POL7080), which specifically targets *P. aeruginosa*, including multidrug-resistant clinical isolates (33). Thus, it could be used for the treatment of antibiotic-resistant *P. aeruginosa* skin infection (34, 35). Given that HDPs including protegrin-1 activate human MCs *via* MRGPRX2 (22, 23, 29), raises the interesting possibility that potential therapeutic action of murepavadin for *P. aeruginosa* skin infection likely reflects both MRGPRX2-mediated MC activation and its direct antimicrobial activity. However, the possibility that murepavadin activates MCs has not been tested.

Besides G proteins, most GPCR agonists activate another signaling pathway that requires the recruitment of adapter proteins known as β-arrestins. This β-arrestin-mediated pathway was first identified for its role in receptor desensitization (uncoupling of receptor/G protein interaction) and internalization (36). Agonists that prefer to activate G proteins over β-arrestins are known as G protein-biased agonists, whereas agonists that selectively activate β-arrestins are known as β-arrestin-biased agonists. By contrast, agonists that activate both pathways are designated as balanced agonists. We have recently shown that while compound 48/80 (C48/80) acts as a balanced agonist for MRGPRX2, an angiogenic host defense peptide serves as a G protein-biased agonist (37). The purpose of this study was to test if murepavadin activates human MCs *via* MRGPRX2 and to determine if it serves as a balanced or biased agonist for the receptor. The data presented herein demonstrate that murepavadin activates human and murine MCs *via* MRGPRX2 and MrgprB2, respectively and that it serves as a G protein-biased agonist for MRGPRX2 without the involvement of β-arrestin-mediated receptor regulation. These findings have important implications for the potential utilization of murepavadin in modulating antibiotic-resistant cutaneous infections.

## Materials and Methods

### Materials

All reagents used for cell culture were purchased from Invitrogen (Gaithersburg, MD, USA). Recombinant mouse interleukin-3 (IL-3), mouse stem cell factor (SCF), and recombinant human SCF (rhSCF) were obtained from Peprotech (Rocky Hill, NJ, USA). Compound 48/80 (C48/80) was obtained from AnaSpec (Fremont, CA, USA). Murepavadin (Catalog HY-P1674A) was from MedChem Express. P-nitrophenyl-N-acetyl-β-D-glucosamine (PNAG) was purchased from Sigma-Aldrich (St. Louis, MO, USA). Pertussis toxin (PTx) was from List Biological Laboratories (Campbell, CA, USA). Fura-2 acetoxymethyl ester was from Abcam (Cambridge, MA, USA). Bright-Glo Luciferase was from Promega (Madison, WI, USA). Phycoerythrin (PE)-conjugated anti-human MRGPRX2 antibody was from BioLegend (San Diego, CA, USA). Amaxa Nucleofector Kit V was from Lonza (Gaithersburg, MD, USA). DuoSet ELISA kits were from R&D Systems (Minneapolis, MN, USA). Hemagglutinin (HA)-tagged MRGPRX2 plasmid in pReceiver-MO6 vector was obtained from GeneCopoeia (Rockville, MD, USA). MRGPRX2-Tango plasmid (Addgene no. 66440) was a gift from Dr. Bryan Roth.

### Mice

C57BL/6 (wild-type; WT) mice were purchased from the Jackson Laboratory (Bar Harbor, ME, USA) and housed in pathogen-free cages. WT mice with the deletion of *MrgprB2* transcript (MrgprB2^-/-^ mice) were generated as previously described (38). Eight-to-twelve-week-old male and female mice were used. All animal experiments performed in this study were approved by the Institutional Animal Care and Use Committee of the University of Pennsylvania.

### Cell Culture

The human MC line (LAD2 cell) was kindly provided by Drs. Kirshenbaum and Metcalfe (Laboratory of Allergic Diseases, National Institute of Allergy and Infectious Diseases, National Institutes of Health (NIH), USA). LAD2 cells were cultured in complete StemPro-34 medium supplemented with l-glutamine (2 mM), penicillin (100 IU/mL), streptomycin (100 μg/mL), and rhSCF (100 ng/mL), and the medium was hemi-depleted weekly (39).

Rat basophilic leukemia (RBL-2H3) cells were cultured as monolayers in Dulbecco’s modified Eagle’s medium (DMEM) supplemented with 10% FBS, L-glutamine (2 mM), penicillin (100 IU/mL) and streptomycin (100 μg/mL) (40). RBL cells stably expressing human MRGPRX2 were maintained similarly in the presence of 1 mg/mL G418. HTLA cells (HEK-293T cells stably expressing a tTA-dependent luciferase reporter and a β-arrestin2-TEV protease fusion gene) were cultured in DMEM supplemented with 10% FBS, L-glutamine (2 mM), penicillin (100 IU/mL), streptomycin (100 μg/mL), hygromycin (200 μg/mL), puromycin (5 μg/mL), and G418 (500 μg/mL) (41). All cell cultures were kept at 37°C incubator with 5% CO_2_.

Peritoneal mast cells (PMCs) were established from peritoneal lavages of WT and MrgprB2^-/-^ mice and were cultured for 4–8 weeks in Iscove’s Modified Dulbecco’s Medium (IMDM) supplemented with 10% FCS, and recombinant mouse IL-3 (10 ng/mL) and SCF (30 ng/mL). Cells were then determined for MC receptor expression and function, and were used within 4–8 weeks (38, 42).

### Degranulation

Human LAD2 (1 x 10^4^ cells/well), RBL-2H3, RBL-MRGPRX2 (5 × 10^4^ cells/well), or murine peritoneal MCs (5 × 10^3^ cells/well) were washed and plated in a total volume of 50 μL HEPES buffer in 96-well plates. Cells were then stimulated with murepavadin for 30 min at 37°C. Total level of β-hexosaminidase release were assessed by lysing the cells with 0.1% Triton X-100, whereas cells without any stimulation were designated as controls. Aliquots (20 μL) of supernatants were incubated with 1 mM PNAG (20 μL) for 1 h at 37°C. The reaction was then stopped by adding stop buffer (250 μL; 0.1 M Na_2_CO_3_/0.1 M NaHCO_3_). Quantification of β-hexosaminidase level was determined by measuring the absorbance at 405 nm using a Versamax microplate spectrophotometer (Molecular Devices, San Jose, CA, USA) (40).

In some experiments, cells were pretreated with PTx (100 ng/mL, 16 h) prior to any stimulation to assess the inhibitory effect of PTx on MC degranulation.

### Calcium Mobilization

Human LAD2 cells (3 × 10^5^), RBL-2H3 or RBL-MRGPRX2 (2 × 10^6^) were loaded with Fura-2 acetoxymethyl ester (1 μM for 30 min at 37°C) in 1.5 mL of HEPES buffer containing 0.1% BSA. Cells were then washed and allowed complete de-esterification for 15 min at room temperature. Cells were then resuspended in buffer and stimulated with Murepavadin or C48/80. Calcium mobilization was determined by the ratio between dual excitation wavelengths of 340 and 380 nm, and an emission wavelength of 510 nm using a Hitachi F-2700 Fluorescence Spectrophotometer.

### Cytokine and Chemokine Production and Measurement

LAD2 cells (3 × 10^5^ cells/mL) were washed with medium, resuspended in fresh medium, and stimulated with indicated concentrations of Murepavadin for 24 h at 37°C with 5% CO_2_. Cell-free supernatants were collected and kept at -80°C until further analyses. Similarly, RBL-2H3 or RBL-MRGPRX2 cells (2 × 10^5^ cells/mL) were seeded in a 24-well plate and cultured overnight in a 37°C incubator with 5% CO_2_. The next day, the medium was aspirated, fresh medium was added to the cells, and the cells were stimulated with indicated concentrations of Murepavadin for 24 h at 37°C with 5% CO_2_. Cell-free supernatants were collected and kept at -80°C until further analyses. The cytokine and chemokine production were measured using human CCL3/MIP-1 alpha, human IL-8/CXCL8, rat JE/MCP-1/CCL2 and rat TNF-alpha DuoSet ELISA kits (R&D Systems) following the manufacturer’s protocols.

To determine the inhibitory effect of PTx on cytokine and chemokine production, pretreatment with PTx (100 ng/mL, 16 h) was performed prior to any stimulation.

### Generation of Cells Transiently Expressing MRGPRX2 and Its Variants

Transient transfections in RBL-2H3 cells expressing WT-MRGPRX2 and its naturally occurring missense variants within MRGPRX2’s ligand binding cradle (G165E) or G protein-coupling region (V282M) were performed as described previously (43, 44). RBL-2H3 cells (2 × 10^6^) were transfected with 2 µg of HA-tagged plasmid using the Amaxa Nucleofector Device and Amaxa Kit V and were used within 16 – 20 h post-transfection.

Flow cytometry was used to determine cell surface expression of transiently transfectants. Cells (5 × 10^5^) were incubated with PE-anti-MRGPRX2 antibody for 30 min, washed in ice-cold FACS buffer (PBS containing 2% FCS and 0.09% NaN_3_), followed by fixation with 1.5% paraformaldehyde. Expression level of MRGPRX2 and its variants were analyzed using a BD LSR II flow cytometer (San Jose, CA, USA) with WinList software, version 8.

### Transcriptional Activation Following Arrestin Translocation (Tango) Assay

HTLA-MRGPRX2 cells (5 × 10^4^ cells/well, 96-well plate) were cultured overnight in a 37°C incubator. The next day, the medium was removed and cells were exposed to Murepavadin in an antibiotic-free medium (160 μL) for 16 h at 37°C. The medium was then replaced with 100 μL of Bright-Glo solution and relative luminescence was analyzed using a Thermo Luminoskan Ascent 392 Microplate Luminometer (41).

### Receptor Internalization

RBL-MRGPRX2 or HTLA-MRGPRX2 cells (5 × 10^5^) were treated with C48/80 or Murepavadin for 30 min, 3, 6, and 16 h to induce cell surface receptor internalization. After indicated time, cell surface expression was determined by flow cytometry as described above.

### Evan’s Blue Dye Extravasation

Mice (WT and MrgprB2^-/-^) were intravenously injected with 1% Evan’s blue followed by intradermal injection of 20 µL Murepavadin (30 µM) in the right paw and PBS (vehicle) in the left paw. After 30 min, the mice were euthanized and the paws were removed, weighed, dissolved in 500 µL formamide and incubated at 56°C overnight. The Evan’s blue dye extravasation was measured by collecting the supernatants and the absorbance was measured at 650 nm using microplate spectrophotometer.

### Statistical Analysis

Data shown represent mean ± SEM value derived from at least three independent experiments. Statistical significance was calculated using *t*-test and one-way or two-way ANOVA analyzed by GraphPad Prism version 9.0.1. Significant differences were set at *p < 0.05, **p < 0.01, ***p < 0.001, ****p < 0.0001.

## Results

### Murepavadin Induces Intracellular Cas^2+^ Mobilization, Degranulation and Chemokine Generation in Human MCs

We previously demonstrated that LL-37, human β-defensins and protegrin-1 activate human MCs *via* MRGPRX2 at concentrations ranging from 1 - 10 µM (22, 23, 29). To determine if murepavadin activates MCs, we initially utilized a human MC line, LAD2 cells and tested the ability of 10 µM murepavadin to induce Ca^2+^ mobilization. As shown in **Figure 1A**, murepavadin at this concentration induced a robust and sustained Ca^2+^ response. Next, we asked if murepavadin induces MC degranulation. We found that murepavadin induced a dose-dependent degranulation as measured by β-hexosaminidase release, reaching ~80% at a concentration of 10 μM with an EC_50_ value of ~3 µM (**Figure 1B**). While MC degranulation promotes increased vascular permeability *in vivo*, its innate and adaptive immune function require the generation of chemokines. We therefore investigated the ability of murepavadin to stimulate chemokine IL-8 and CCL3 production in LAD2 cells. At a concentration of 10 µM, murepavadin induced substantial IL-8 (**Figure 1C**) and CCL3 (**Figure 1D**).

**Figure 1:** Murepavadin induces intracellular Ca^2+^ mobilization, degranulation and causes chemokine production in human MCs. **(A)** Ca^2+^ mobilization measurement following murepavadin (10 μM) stimulation of Fura-2-loaded LAD2 cells. **(B)** LAD2 cells were exposed to indicated concentrations of murepavadin (30 min) and degranulation was assayed by measuring the release of β-hexosaminidase. **(C, D)** LAD2 cells were exposed to 10 μM of murepavadin for 24 h and the production of IL-8 and CCL3 were determined by ELISA. Data presented are the mean ± SEM of at least three experiments. Statistical significance was determined by *t*-test or one-way ANOVA with Dunnett’s multiple comparisons at a value **p < 0.01, ***p < 0.001, and ****p < 0.0001.

To explore the underlying mechanism *via* which murepavadin activates MCs, we utilized RBL-2H3 cells that were transfected to stably express human MRGPRX2 (RBL-MRGPRX2). We found that murepavadin induced Ca^2+^ mobilization, β-hexosaminidase as well as TNF-α and CCL2 production from RBL-MRGPRX2, but not from untransfected cells (**Figures 2A–E**). Moreover, we found that Pertussis toxin (PTx), an inhibitor of Gαi/o family of G proteins, caused significant inhibition of murepavadin-induced degranulation, TNF-α and CCL2 production (**Figures 2C–E**). Taken together, these findings demonstrate that murepavadin causes the activation of human MCs specifically *via* MRGPRX2 and that these responses are G protein-dependent.

**Figure 2:** Murepavadin induces intracellular Ca^2+^ mobilization, degranulation and chemokine production in MCs through MRGPRX2. **(A)** Calcium mobilization measurement following murepavadin (10 μM) stimulation of Fura-2 loaded WT-RBL and RBL-MRGPRX2 cells. **(B)** WT-RBL and RBL-MRGPRX2 cells were exposed to 10 μM murepavadin (30 min), and degranulation was assayed by measuring the release of β-hexosaminidase. **(C)** RBL-MRGPRX2 cells were incubated in the presence or absence of pertussis toxin (PTx), at a concentration of 100 ng/mL for 16 h and exposed to indicated concentrations of murepavadin (30 min) and degranulation was assayed by measuring the release of β-hexosaminidase. **(D, E)** WT-RBL and RBL-MRGPRX2 cells were incubated in the presence or absence of pertussis toxin (PTx) at a concentration of 100 ng/mL for 16 h and exposed to 10 μM of murepavadin (24 h) and the production of cytokine TNF-α and chemokine CCL2 were quantified by ELISA. Data presented are the mean ± SEM of at least three experiments. Statistical significance was determined by two-way ANOVA with Šídák’s or Tukey’s multiple comparisons at a value *p < 0.05, ***p < 0.001, ****p < 0.0001, and ns denotes “not significant”.

### Naturally Occurring MRGPRX2 Missense Variants Are Hypo-Responsive to Murepavadin for MC Degranulation

We have previously identified naturally occurring loss-of-function MRGPRX2 missense variants within the receptor’s ligand binding (G165E) and G protein coupling (V282M) domains (**Figures 3A, B** **)** (43, 44). To further validate murepavadin’s specificity for MRGPRX2, we transiently transfected RBL-2H3 cells with cDNAs encoding each of these variants. Flow cytometry analyses confirmed cell surface expression of MRGPRX2 (WT) and its missense variants (G165E and V282M) (**Figure 3C**). While murepavadin (10 µM) induced β-hexosaminidase release in cells expressing WT-MRGPRX2, this response was significantly inhibited in cells transiently expressing the G165E or V282M variant (**Figure 3D**). These findings substantiate the notion that murepavadin utilizes MRGPRX2 to activate MCs.

**Figure 3:** Naturally occurring MRGPRX2 missense variants are hypo-responsive to murepavadin for MC degranulation. **(A)** Snake diagram of MRGPRX2 indicating the two amino acid residues to be investigated. **(B)** Single amino acid substitution for each of the MRGPRX2 variant is shown in the table. **(C)** Cell surface receptor expression of the wild-type MRGPRX2 (WT) and its missense variants (G165E and V282M) was confirmed using flow cytometry. **(D)** RBL cells expressing MRGPRX2 (WT) and its variants (G165E and V282M) were exposed to 10 μM murepavadin (30 min) and degranulation was assayed by measuring the release of β-hexosaminidase. Statistical significance was determined by two-way ANOVA with Tukey’s multiple comparisons at a value **p < 0.01 and ****p < 0.0001.

### Murepavadin Does Not Promote β-Arrestin Recruitment Following MRGPRX2 Activation

To determine if murepavadin promotes β-arrestin recruitment in addition to G proteins, we utilized HTLA (HEK-293T cells that were transfected with a tTA-dependent luciferase reporter and a β-arrestin2-TEV protease fusion gene) cells stably expressing MRGPRX2 (HTLA-MRGPRX2). We have previously shown that C48/80 strongly promotes β-arrestin recruitment in HTLA-MRGPRX2 cells as determined by a transcriptional activation following arrestin translocation (Tango) assay (37). We therefore utilized C48/80 as a positive control and tested the ability of murepavadin to promote β-arrestin recruitment. As shown in **Figures 4A, B**, while C48/80 (3 µg/mL) induced ~30-fold increase in β-arrestin-mediated gene expression when compared to buffer control, murepavadin was without effect.

**Figure 4:** Murepavadin does not promote β-arrestin recruitment following MRGPRX2 activation. **(A, B)** HTLA-MRGPRX2 cells were exposed to indicated concentrations of C48/80 or murepavadin for 16 h. Medium was removed and Bright-Glo solution (100 µL) was added into each well (96-well plate) and β-arrestin gene expression (in relative luminescence unit) was measured. **(C, D)** HTLA-MRGPRX2 cells were exposed to MRGPRX2 ligand (C48/80 or murepavadin, 16 h) and cell surface receptor expression of MRGPRX2 was confirmed using flow cytometry and quantified using a mean fluorescent intensity (MFI) in comparison to the untreated control. **(E, F)** Representative histograms of MRGPRX2 cell surface receptor expression of HTLA-MRGPRX2 cells. Statistical significance was determined by one-way ANOVA with Dunnett’s multiple comparisons at a value ****p < 0.0001 and ns denotes “not significant”.

### Murepavadin Does Not Induce MRGPRX2 Internalization or Desensitization

We have previously shown that C48/80 not only induces β-arrestin recruitment but also causes MRGPRX2 internalization (37). We found that incubation of HTLA-MRGPRX2 cells with C48/80 (3 µg/mL; 0.5 h -16 h) induced substantial receptor internalization but murepavadin had no effect **(** **Figures 4C, D** **)**. The data presented in **Figures 4E, F** show representative histograms of cell surface MRGPRX2 following incubation of HTLA-MRGPRX2 cells with C48/80 (3 µg/mL) and murepavadin (10 µM) for 16 h. These data clearly demonstrate that while C48/80 promotes β-arrestin recruitment and caused MRGPRX2 internalization, murepavadin does not induce these responses.

To confirm the biological relevance of the findings described above, we performed receptor internalization studies in RBL-MRGPRX2 cells by flow cytometry. Similar to the situation in HTLA-MRGPRX2 cells, C48/80 induced substantial receptor internalization in RBL-MRGPRX2 cells but murepavadin had no effect (**Figures 5A, B** **)**. As for β-arrestin recruitment (**Figure 4A**) and receptor internalization (**Figures 5A, B** **)**, incubation of cells with C48/80 (3 µg/mL, 16 h) resulted in substantial inhibition of Ca^2+^ mobilization response to the stimulation by the same agonist (**Figure 5C**). Conversely, cells preincubated with murepavadin (10 µM, 16 h) had little to no effect on Ca^2+^ response to stimulation by the same agonist (**Figure 5D**).

**Figure 5:** Murepavadin does not induce MRGPRX2 internalization or desensitization. **(A)** RBL-MRGPRX2 cells were exposed to MRGPRX2 ligand (C48/80 3 μg/mL or murepavadin 10 μM, 16 h) and cell surface receptor expression of MRGPRX2 was confirmed using flow cytometry. A representative histogram of MRGPRX2 cell surface receptor expression is shown. **(B)** Quantitative analysis of cell surface receptor expression was calculated using a mean fluorescent intensity (MFI) in comparison to the untreated control. **(C, D)** Calcium mobilization measurements of RBL-MRGPRX2 cells exposed to MRGPRX2 ligand (C48/80 3 μg/mL or murepavadin 10 μM, 16 h) following C48/80 (3 μg/mL) or murepavadin (10 μM) stimulation, respectively. Statistical significance was determined by one-way ANOVA with Dunnett’s multiple comparisons and two-way ANOVA with Šídák’s multiple comparisons at a value *p < 0.05, **p < 0.01, ***p < 0.001, ****p < 0.0001, and ns denotes “not significant”.

### Murepavadin Activates Murine MCs *In Vitro* and *In Vivo via* MrgprB2

It has been previously shown that C48/80 causes substantial degranulation in mouse peritoneal MCs (PMCs) *via* MrgprB2 (21). To test if murepavadin induces degranulation in murine PMCs and to determine the role of MrgprB2 in this response, we cultured PMCs from peritoneal lavage of wild-type (WT) and MrgprB2^-/-^ mice (38, 42). We found that murepavadin induced degranulation in PMCs cultured from WT mice but this response was not observed in cells cultured from MrgprB2^-/-^ mice (**Figure 6A**). To determine if murepavadin induces degranulation of cutaneous MC *in vivo*, we performed intradermal injection of murepavadin (30 µM, 20 µL) or PBS into the paw after intravenous injection of Evan’s blue dye. Consistent with peritoneal MC degranulation *in vitro*, murepavadin caused a significant increase in vascular permeability when compared to PBS. However, this vascular permeability response was abolished in MrgprB2^-/-^ mice (**Figures 6B, C** **)**. Together, these data demonstrate that murepavadin induces degranulation in murine MCs to cause increased vascular permeability *via* the activation of MrgprB2.

**Figure 6:** Murepavadin activates murine MCs *in vitro* and *in vivo via* MrgprB2. **(A)** WT and MrgprB2**^-/-^** PMCs were exposed to 10 μM murepavadin (30 min) and degranulation was assayed by measuring the release of β-hexosaminidase. **(B)** Representative images of Evan’s blue dye extravasation in WT and MrgprB2**^-/-^** mice *in vivo.* Mice were intradermally injected with 20 μL of murepavadin (30 μM) or PBS, and extravasation of Evan’s blue dye was determined after 30 min. **(C)** Quantification of extravasation of Evan’s blue dye in WT and MrgprB2**^-/-^** mice (n = 7-8). Statistical significance was determined by two-way ANOVA with Tukey’s multiple comparisons at a value **p < 0.01, ***p < 0.001, ****p < 0.0001, and ns denotes “not significant”.

## Discussion

Murepavadin is a synthetic cyclic β-hairpin HDP mimetic that targets an outer membrane protein transporter LptD of the Gram-negative bacterium *P. aeruginosa*, which makes it highly specific to this pathogen (45, 46). In *in vitro* studies, murepavadin is very effective against a wide-ranging species of multi-drug resistant *Pseudomonas* bacteria and demonstrates exceptional efficacy in sepsis, lung, and thigh infection models *in vivo* (47). However, intravenous administration of murepavadin for treating nosocomial pneumonia has been temporarily halted due to reports of kidney injury. Despite this, an inhaled formulation of murepavadin is under investigation for its potential effectiveness in treating *Pseudomonas* infection in patients with cystic fibrosis (33, 48). We made the novel observation that murepavadin is able to induce human MC activation through MRGPRX2 and murine MC activation through MrgprB2. Because human skin MCs express MRGPRX2 at high levels (17, 19, 49), these findings suggest that murepavadin can be utilized for treating *P. aeruginosa* skin infection through harnessing MC’s host defense and wound healing properties.

*P. aeruginosa* skin infection is associated with high morbidity and mortality rates mainly because of its ability to form biofilms and to resist multiple antibiotics (25, 26). Therefore, novel treatment approach together with rapid wound closure are critical to control this type of infection. Weller et al. (50), showed that skin wounding in mice results in MC degranulation. This, in turn, causes increased vascular permeability and neutrophil recruitment. Using the same wound model but superimposed with *P. aeruginosa*, Zimmerman et al. (27), showed that MCs are essential in controlling bacterial infection and promoting healing. It was proposed that IL-1 and IL-33 generated by keratinocytes in response to infection activate MCs to produce IL-6, which in turn generate HDPs from keratinocytes resulting in the direct bacterial killing. However, recent studies demonstrated that HDPs can also induce MC degranulation in human (*via* MRGPRX2) and mouse (*via* MrgprB2) (22–24). Based on these findings, we suspect that the activation of MCs *via* MRGPRX2/B2 confer protective immunity and contribute to host defense. The minimum concentration of murepavadin required to inhibit 90% growth of *P. aeruginosa* (MIC_90_) was reported to be in the range of 2 - 32 mg/L (33, 48). We found that murepavadin (1 µM; 1.667 mg/L) induced significant MC degranulation *via* MRGPRX2 and that maximal response was obtained at a concentration of 10 µM (16.67 mg/L). Murepavadin at 10 µM, which is relevant for direct inhibition of *P. aeruginosa* growth, induced TNF-α, IL-8 and CCL3 production from MCs *via* MRGPRX2. A topical application of murepavadin is currently under investigation for treating *P. aeruginosa* cutaneous infection mainly because of its direct and specific activity against the pathogen (34, 35). Based on the data presented herein, we propose that potential effectiveness of murepavadin also reflects its ability to harness MC’s immunomodulatory property *via* the activation of MRGPRX2 (**Figure 7**).

**Figure 7:** Proposed mechanism of action of murepavadin/MRGPRX2-induced bacterial clearance and wound healing. Murepavadin activates MCs *via* MRGPRX2. An increase in intracellular calcium following murepavadin stimulation triggers MC degranulation and chemokine production (IL-8, CCL3, CCL2, and TNF-α). These MC mediators induce immune cell recruitment and subsequently contribute to host defense and wound healing.

It is well documented that *Staphylococcus aureus* is responsible for the majority of bacterial skin infections (51, 52). In a murine model of *S. aureus* skin infection, topical application of mastoparan, an amphipathic peptide found in *Hymenoptera* venom that causes MC activation *via* MrgprB2, results in the recruitment of immune cells particularly neutrophils, This contributes to subsequent bacterial clearance (15). However, a mastoparan derivative that does not induce MC degranulation is unable to control *S. aureus* infection despite the fact that it demonstrates direct antibacterial activity. By contrast, another mastoparan derivative that induces MC degranulation *via* MrgprB2 but has no direct antibacterial activity effectively controls infection. These findings suggest that the potential therapeutic effectiveness of mastoparan could reflect its action on MCs *via* MRGPRX2 rather than its direct antibacterial activity.

Apart from degranulation, mastoparan also triggers the generation of chemokines CCL2, CCL3 and CCL4 from MCs, which promote the mobilization of dendritic cells (DCs) including CD301b^+^ dermal dendritic cells (DDCs). DDCs have been implicated in promoting re-epithelialization of sterile wounds and accelerating wound closure. Depletion of MrgprB2-expressing MCs results in significantly decreased number of DDCs, suggesting that MCs contribute to the restoration of DDCs population to homeostatic levels, thus contributing to regenerative healing (15). Moreover, mastoparan also contributes to the production of *S. aureus*-specific IgG following initial *S. aureus* skin infection, which is associated with reduced lesion size during subsequent bacterial reinfection (15). Thus, it is highly likely that activation of murine MCs by mastoparan through MrgprB2 confers both innate and adaptive immunity to provide protection against bacterial infection and reinfection. Given that murepavadin activates human MCs *via* MRGPRX2, it should be possible to use this HDP mimetic for the modulation of *S. aureus* skin infection. Because murepavadin appears to have a lower EC_50_ value for MC degranulation than mastoparan (15), our prediction is that lower concentration of the drug will be required to treat *S. aureus* infection. Also, since murepavadin is an HDP mimetic and is less susceptible to degradation than mastoparan, its effectiveness is likely to be greater than that of mastoparan, thus requiring fewer treatments to clear infection and to promote healing.

It is generally accepted that most GPCRs activate two parallel but independent signaling pathways; one involving G proteins while second pathway is independent of G proteins but requires the recruitment of β-arrestins (53–56). For certain GPCRs, agonists can activate only G proteins (G protein biased) or only β-arrestin (β-arrestin biased) or both (balanced). Agonists that induce both pathways not only activate G protein-mediated signaling but also result in dissociation of G proteins from the receptor (desensitization) and promote the receptor internalization. We have previously shown that while C48/80 acts as balanced agonist for MRGPRX2, an HDP angiogenic peptide, AG-30/5C acts as a G protein-biased agonist for the receptor. Thus, C48/80 caused substantial β-arrestin recruitment while AG-30/5C had little to no effect. Most importantly, preincubation of cells with C48/80 resulted in a significant reduction of cell surface receptor expression and loss of cell responsiveness to all MRGPRX2 agonists tested. By contrast, AG-30/5C had little to no effect on cell surface receptor expression or MC degranulation to any of the MRGPRX2 agonists tested (37). The data presented herein demonstrate that similar to AG-30/5C, murepavadin acts as a G protein-biased agonist for MRGPRX2. Thus, it is possible that the resistance MRGPRX2 to undergo desensitization and internalization by murepavadin could enhance its therapeutic potential.

In summary, although HDPs have therapeutic potential for the treatment of multi-drug-resistant bacterial infections, their relative instability and cytotoxicity have limited their usefulness as prospective antimicrobial agents. Small molecule HDP mimetics do not display these limitations and murepavadin was synthesized to specifically target *P. aeruginosa.* However, the possibility that murepavadin could activate MCs has not been suspected. In the present study, we have shown that murepavadin induces degranulation, TNF-α, IL-8 and CCL3 production *via* MRGPRX2, a receptor that is primarily expressed in human skin MCs. Thus, the ability of murepavadin to exploit MC’s immunomodulatory functions could form the basis for the treatment of skin infection caused by bacterial species such as *P. aeruginosa* and *S. aureus.* Furthermore, the findings presented herein that MCs expressing missense MRGPRX2 variants G165E (rs141744602) and V282M (rs779414608) were resistant to murepavadin-induced degranulation likely has important clinical implications. It is possible that murepavadin may not effectively clear microbial infection in individuals harboring these MRGPRX2 polymorphisms because of their inability to support MC degranulation.

## Data Availability Statement

The original contributions presented in the study are included in the article/supplementary material. Further inquiries can be directed to the corresponding author.

## Ethics Statement

The animal study was reviewed and approved by The Institutional Animal Care and Use Committee of the University of Pennsylvania.

## Author Contributions

HA contributed to conception, supervision and funding acquisition of the study. AA and CC performed the experiments and analyzed the data. AA and HA wrote the first draft of the manuscript. All authors contributed to the article and approved the submitted version.

## Funding

This work was supported by grants R01-AI143185, R01-AI149487 and R01-AI124182 to HA.

## Conflict of Interest

The authors declare that the research was conducted in the absence of any commercial or financial relationships that could be construed as a potential conflict of interest.
